# Negative Regulation of Tec Kinase Alleviates LPS-Induced Acute Kidney Injury in Mice via theTLR4/NF-*κ*B Signaling Pathway

**DOI:** 10.1155/2020/3152043

**Published:** 2020-06-19

**Authors:** Wei Zhang, Ping Zhou, Xiao Jiang, Zhe Fan, Xingxin Xu, Fei Wang

**Affiliations:** ^1^Department of Nephrology, The First Affiliated Hospital of Anhui Medical University, Hefei, Anhui 230022, China; ^2^Department of Burns, The First Affiliated Hospital of Anhui Medical University, Hefei, Anhui 230022, China

## Abstract

Tec kinase is an important mediator in inflammatory immune response that enhances the activity of neutrophils and macrophages. However, information on its function in lipopolysaccharide- (LPS-) induced acute kidney injury (AKI) is limited. This study is aimed at determining whether Tec kinase was a regulator in AKI. An AKI model in mice was successfully established using intraperitoneal LPS. Results showed that the serum levels of creatinine (Cr), blood urea nitrogen (BUN), and cystatin-C (Cys-C) increased after intraperitoneal LPS injection. Renal tissue sustained significantly severe injury as measured by pathological scores. Pretreatment with LFM-A13 improved the function of the kidney in mice and decreased the renal injury score. Enzyme-linked immunosorbent assay showed that LFM-A13 significantly reduced the release of IL-1*β* and TNF-*α* in mice exposed to LPS. LFM-A13 can evidently abrogate the expression of Tec protein, MyD88, TLR4, NF-*κ*B p65, and Tec's phosphorylated protein as determined by Western blot. Immunohistochemistry analysis revealed that LFM-A13 markedly downregulated the expression of Tec kinase in renal tubular epithelial cells. In vitro, Tec kinase protein was expressed highly in NRK-52E cells after LPS exposure. Tec-siRNA also decreased IL-1*β* and TNF-*α* production and obviously abolished phospho-p65 and phospho-I*κ*B*α* expression in NRK-52E cell stimulated by LPS; however, Tec-siRNA increased the I*κ*B*α* level. Altogether, these data suggested that Tec kinase can be a modulating protein in AKI through TLR4/NF-*κ*B activation.

## 1. Introduction

Sepsis is a heterogeneous clinical syndrome that is broadly defined as a systemic inflammatory response to infection, which causes multiple organ dysfunction including the kidney. Acute kidney injury (AKI) is a common kidney disorder associated with high morbidity and mortality rates, especially in critically ill patients [1, 2]. AKI is a well-defined and independent risk factor of mortality in all septic patients, accounting for approximately 70% [3, 4]. The pathogenesis of AKI in sepsis is complex and caused by multiple or many factors, including inadequate vascular leakage/perfusion, local tubular inflammation, and renal endothelial dysfunction [5–7]. Among these factors, the early inflammation responses in kidneys are increasingly recognized as a major mechanism of sepsis-induced AKI. Previous studies have indicated that endotoxins, such as lipopolysaccharide (LPS), bind to Toll-like receptor 4 (TLR4), leading to the activation of the NF-*κ*B pathway in septic AKI, and these processes are initiated a few hours with the production of cytokines, such as TNF-a and IL-1, and the infiltration and activation of immune cells [8, 9]. Castoldi et al. reported that TLR2, TLR4, and MyD88 mRNAs are highly expressed in the renal tissue after sepsis. IL-1*β* and TNF-*α* production decreased, and the NF-*κ*B p65 translation to the nucleus was inhibited in TLR2-/-, TLR4-/-, and MyD88-/- mice because of improved kidney function [10].

Tec is a nonreceptor tyrosine kinase that is initially found in hepatocellular carcinoma. Tec family kinases, such as Bmx, Btk, Itk, and Tec, are phosphorylated and activated in the early stages of the inflammatory response [11–13]. The mechanism of Tec kinase in inflammatory response to sepsis in neutrophils and macrophages was recently studied. Tampella et al. showed that primary resident peritoneal macrophages deficient in Tec kinase secrete less proinflammatory cytokines, such as IL-6 and TNF-*α*, in response to the TLR stimulation of LPS (TLR4 ligand) and Pam3CKS4 (TLR1/2 ligand) relative to the cells isolated from wild-type mice [14]. Zemans and Arndt considered Tec kinase as an upstream component of the signaling pathway that leads to LPS-induced MAPK activation in neutrophils [15]. Our previous works also suggested that LPS induces the phosphorylation of Tec kinase in RAW264.7 cells, and inhibition of Tec kinase by LFM-A13 or siRNA decreases monocyte chemotactic protein- (MCP-) 1 secretion and the intercellular adhesion molecule- (ICAM-) 1 expression [16]. However, whether Tec kinase has any role in regulating tissue damage after AKI is unclear.

In this study, we used a sepsis-induced AKI mouse model to investigate the Tec kinase expression. Meanwhile, the suppression of Tec kinase by LFM-A13 pretreatment in vivo and Tec siRNA transfection in vitro was attempted to elucidate the inflammatory effect of Tec kinase on AKI. To explore the underlying mechanisms further, the involvement of NF-*κ*B and upstream protein, such as TLR4 and MyD88, was also assessed.

## 2. Materials and Methods

### 2.1. Animals and Groups

Adult C57BL/6 mice were purchased from the Experimental Animal Center of Anhui Medical University. Male mice weighing 22-26 g were used for the experiments. They were housed under specific pathogen-free (SPF) conditions for one week. All the animals were sterile. The drinking water, pad, and feed were sterilized by high-pressure boiling subjected to identical antiseptic treatments. The relative humidity, the temperature, and the illumination of the rearing room were 50%-55%, 20°C, and 12 h. Animal experiments conform to the regulations of the Anhui Province on the administration of laboratory animals. All procedures were performed in accordance with the ethical standards for the use and care of animals. On the following day, 32 mice were randomly assigned to two groups (*n* = 16). LPS (Sigma, St. Louis, MO) (20 mg/kg, 1 mg/mL in 0.9% normal saline) was intraperitoneally injected in the LPS group of mice, and an equal dose of solvent was injected in the control group. No deaths were recorded among the experimental mice. At 1, 6, 24, and 48 h, 4 mice from each group were sacrificed. To investigate the effect of LFM-A13 (Tocris Biosciences), we randomly divided the other 36 mice into 6 groups (*n* = 6). The LPS group received an intraperitoneal injection of LPS 20 mg/kg, and the control group was given the same amount of solvent. LFM-A13 doses (40, 60, and 80 mg/kg) were administered i.p. immediately after LPS exposure. The peritoneal perfusion fluid volume of mice was 1 mL/20 g. The mice were sacrificed and perfused at 24 h.

### 2.2. Cell Culture and Reagents

Mouse renal tubular epithelial cell line NRK-52E cells was obtained from the Chinese Type Culture Collection (Shanghai Institute of Cell Biology, China) and were inoculated in a sterile culture flask containing calf serum high-glucose DMEM at 37°C in a humidified atmosphere of 5% CO_2_. When growing together like cobblestones, the cells were seeded on 6-well BioFlex collagen-coated culture plates and grown to 80% confluence. The FBS concentration was reduced to 1% 24 hours prior to the experiments. The cells were stimulated with LPS (Sigma, St. Louis, MO) of different concentrations and duration. To study the role of Tec kinase in renal tubular epithelial cells, different concentrations of LFM-A13, a leflunomide metabolite analogue, were added to the cells 1 h before stimulation with LPS.

The reagents used in this study were purchased from the following sources: LFM-A13 from Tocris Bioscience and Tec siRNA from Genepharma Co., Ltd. (Shanghai, China); and all monoclonal antibodies for NF-*κ*B p-p65, p65, I*κ*B*α*, and p-I*κ*B*α* were purchased from Protein Tech Group (Chicago, IL, USA). The antibodies for Tec protein, TLR4, MyD88, and *β*-actin were obtained from Santa Cruz Biotechnology (Santa Cruz, CA).

### 2.3. Biochemical Measurements

Serum was collected from the mice and sent to the clinical laboratory and detected by the Roch Moular D and P automatic biochemical analyzer. Blood urea nitrogen (BUN), serum creatinine (sCr), and cystatin-C (Cys-C) were used for assessing the renal function as important indexes of renal injury severity. The BUN level was detected by the rate method, the sCr level by enzyme colorimetry, and the serum Cys-C level by immunoturbidimetry. Their concentrations were expressed as mmol/L, *μ*mol/L, and mg/L, respectively.

### 2.4. Enzyme-Linked Immunosorbent Assay

The cytokine levels of TNF-*α* and IL-1*β* were measured using a commercially available enzyme-linked immunosorbent assay (ELISA) kit (R&D Systems Europe, Abingdon, United Kingdom) according to the manufacturer's instructions. The TNF-*α* and IL-1*β* protein levels were calculated using the standard curve prepared from sample cytokines. All samples were run in duplicate and averaged.

### 2.5. Western Blot Analysis

Kidney tissue (100 mg) and NRK-52E cells were homogenized in RIPA lysate (containing 10 *μ*L PMSF in RIPA per 1 mL). After incubation on ice for 30 min, the homogenates were centrifuged at 12,000× g for 30 min at 4°C. The resulting supernatant was collected. Protein (25 *μ*g) was mixed with buffer and loaded on 4%-12% SDS-polyacrylamide gradient gels and transferred to a PVDF membrane. After blocking with 5% nonfat milk powder at room temperature for 2 h, the membranes were incubated overnight at 4°C with primary antibodies for Tec (1 : 1000), NF-*κ*B p65 (1 : 1000), phosphorylated p65 (1 : 1000), I*κ*B*α* (1 : 500), phosphorylated I*κ*B*α* (1 : 500), TLR4 (1 : 1000), MyD88 (1 : 1000), and *β*-actin (1 : 1000). Anti-rabbit horseradish peroxidase- (HPR-) conjugated antibody was used as a secondary antibody, and then, all blots were exposed to an enhanced chemiluminescence detection system (Amersham, Little Chalfont, UK). All Western blot analyses were repeated three times.

### 2.6. siRNA Interference

NRK-52E cells were maintained in 75 cm^2^ tissue culture flasks in Dulbecco's modified Eagle's medium (DMEM) supplemented with 10% fetal bovine serum in a humidified 5% CO_2_/95% air incubator at 37°C. According to the Tec gene sequence, an effective siRNA for Tec (sense 5′-GAGGCCAAGAGUAUAUCAUTT-3′ and antisense 5′-AUGAUAUACUCUCGGCCUCTT-3′) was designed and synthesized by Genepharma Co., Ltd. (Shanghai, China). NRK-52E cells were transfected with the negative control siRNA, Tec siRNA using the Lipofectamine 2000 reagent (Invitrogen, Carlsbad, CA) according to the manufacturer's instructions. After incubation for 4 h, the medium was changed with a fresh complete culture medium. The cells were then incubated for an additional 48 h and treated with LPS.

### 2.7. Morphological Analysis

Paraffin-embedded kidney sections were prepared as previously described [17]. Morphological analysis was performed on 3 *μ*m thick sections of paraffin embedded material, stained with hematoxylin and eosin (HE), and examined by light microscopy. Twenty-five consecutive interstitial fields without glomeruli were chosen randomly. The tubulointerstitial injury was evaluated and graded as follows: 0, normal; 1, the area of interstitial inflammation and fibrosis, tubular atrophy and dilation with cast formation involving <25% of the field; 2, lesion area between 25% and 50% of the field; and 3, lesions involving >50% of the field. The tubulointerstitial injury index was blindly evaluated by two renal pathologists according to a semiquantitative criterion [18]. The score was calculated by averaging the grades assigned to all tubule fields.

In immunohistochemistry (IHC) analysis, antigen retrieval was performed in a microwave oven with citrate buffer (pH 6.0) for 10 min. After treatment with 10% calf serum for 10 min, the sections were incubated with primary antibody anti-Tec kinase (1 : 50), at 4°C overnight, The sections were further incubated with HRP-labeled antibody for 20 min at 37°C. Immunostaining was developed by using chromogen 3,3′-diaminobenzidine (DAB, Sigma). All measurements and scoring were performed on blinded slides.

### 2.8. Statistical Analysis

The data were expressed as the means ± standard error of the means (SEMs) and analyzed by one-way analysis of variance (ANOVA), followed by the Student–Newman–Keuls test. Statistical analyses were performed using the SPSS software package (IBM Corporation, Armonk, NY, USA). ^∗^*P* < 0.05 and ^∗∗^*P* < 0.01 were considered statistically significant.

## 3. Results

### 3.1. LPS Injection Intraperitoneally Induces Renal Dysfunction in Mice

The Cr and BUN in serum are usually investigated in AKI. Cys-C is an early predictive biomarker for AKI definition [19]. We evaluated the renal injury measured in terms of serum Cr, Bun, and Cys-C at different times following LPS injection. ELISA analysis showed that the mean serum Cr and BUN levels in LPS-injected mice were significantly higher than those in the control at 24 h (Figures 1(a) and 1(b)). A nonsignificant difference was observed between those groups at 1 h and 48 h. Exposure to LPS resulted in a high level of Cys-C at 6 h that peaked at 24 h and increased to a higher level at 48 h (Figure 1(c)). Subsequently, HE staining was applied to detect the histological changes in renal tissues. Compared with the control, the LPS-induced mass tubule disruption included the vacuolization of tubular cells, loss of brush border, tubular epithelial cell swelling, and interstitial edema (Figure 1(d)). The histology score based on the number of areas with edema, necrosis, and infiltration of inflammatory cells in the renal glomerulus and tubules increased significantly in LPS-exposed mice at the indicated time and peaked at 24 h (Figure 1(e)).

### 3.2. Tec Kinase Is Induced in Mice following LPS Injection Intraperitoneally and LPS-Exposed NRK-52E Cell

As shown in Figures 2(a) and 2(b), compared with the control conditions, LPS injection induced a significant increase in Tec kinase expression and peaks at 1 h and 6 h (*P* < 0.01). Tec kinase protein decreased gradually at 24 and 48 h, but still higher than the sham group (*P* < 0.05). Then, IHC experiment was performed to reveal the localization of Tec kinase in the paraffin sections of renal tissues. Tec kinase was found in the renal tubular epithelial cells of the proximal and distal convoluted tubules in the control. Similar to the Western blot analysis, a maximal Tec kinase expression was markedly detected in the tubular epithelial cells and the interstitium at 1 h (Figure 2(c)). The in vitro NRK-52E cells of the rat kidney proximal tubular epithelial cell line were incubated with various concentrations of LPS (0.01–10 *μ*g/mL) for 1 h. Compared with the control, Tec kinase was significantly induced with a peak expression after the 0.1 *μ*g/mL of LPS treatment (Figure 2(d)). As shown in Figure 2(e), the 0.1 *μ*g/mL of LPS increased the Tec expression in a time-dependent manner, with a peak at 60 min. These results indicated that Tec kinase may be correlated with the development of renal injury.

### 3.3. LFM-A13 Decreases Serum Levels of Cr, BUN, Cys-C, and Pathologic Injury in the Mouse Model of LPS-Induced AKI

We sought to determine the potential role of Tec kinase in renal function and tissue injury. Different concentrations of LFM-A13, a leflunomide metabolite analogue, were used to treat mice prior to LPS injection. As shown in Figures 3(a)–3(c), LPS-treated mice obviously exhibited increased levels of serum Cr, BUN, and Cys-C. However, pretreatment with LFM-A13 (40, 60, and 80 mg/kg) significantly decreased the LPS-induced Cr, BUN, and Cys-C levels in a nondosage-dependent manner. Meanwhile, the histopathological change and the injury score were also evaluated. Renal damage, including focal tubular cell swelling, dilation of renal capsule cavity, and destruction of tubular structures and the epithelial cells of the local focal necrosis collapse, was obviously detected in LPS-injected mice. LFM-A13 pretreatment significantly diminished LPS-induced tubular epithelial necrosis, neutrophil emigration, and interstitial edema. On the basis of the evaluation of the blinded observer, a significant increasing pathological damage score was observed in LPS-treated mice. The inhibitory effect of LFM-A13 was not dosage-dependent (Figures 3(d) and 3(e)).

### 3.4. LFM-A13 Decreases LPS-Induced Tec Protein Expression in Mice after AKI

Next, we examined the effects of LFM-A13 on Tec protein expression on acute tubular injury after LPS injection. As shown in Figure 4(a), IHC staining demonstrated an increased Tec kinase protein in renal tubules after LPS injection compared with controls. The cytoplasmic localization of Tec was evident in renal tubular segments, including proximal tubule and distal tubule, in AKI after LPS i.p. (arrowheads in the boxed area). To confirm this finding, the Western blot analysis of whole kidney lysates was used to assess the renal Tec kinase abundance quantitatively. As illustrated in Figures 4(b) and 4(c), a marked increase in renal Tec protein was observed in LPS-treated mice compared with the controls. Furthermore, the pretreatment of LFM-A13 dose dependently (40, 60, and 80 mg/kg) inhibited the LPS-induced Tec kinase expression. A similar decrease in Tec protein in IHC staining was also apparently detectable in mice pretreated with LFM-A13 prior to LPS injection.

### 3.5. LFM-A13 or Knockdown of Tec by siRNA Decreases LPS-Induced TNF-*α* and IL-1*β* Production in Mice after AKI and in NRK-52E Cell

TNF-*α* and IL-1*β* are important proinflammatory mediators in LPS-induced AKI [20]. The levels of TNF-*α* and IL-1*β* increased significantly after LPS injection intraperitoneally at 24 h compared to those of the control groups (*P* < 0.01, Figure 5), while the pretreatment with LFM-A13 (40, 60, or 80 mg/kg) prior to LPS injection resulted in an obvious decrease in TNF-*α* and IL-1*β* production in a nondose-dependent manner (*P* < 0.05 and *P* < 0.01, respectively). In addition, these cytokines also increased in LPS-stimulated NR-52E cells (data not shown). Accordingly, when NR-52E cells were transfected with siRNA targeting Tec prior to LPS exposure, the release of TNF-*α* and IL-1*β* decreased (data not shown).

### 3.6. LFM-A13 or Knockdown of Tec by siRNA Decreases LPS-Induced TLR4/MyD88/NF-*κ*B Activation in Mice after AKI and in NRK-52E Cell

NF-*κ*B is an important transcription factor in regulating cytokines such as TNF-*α* and IL-1*β* [21]. Thus, we evaluated the effect of LFM-A13 on the expression of NF-*κ*B signals in mice after AKI. To investigate the NF-*κ*B activity in mice, phospho-p65 and p65 were analyzed by Western blot analysis. As shown in Figures 6(a) and 6(b), the intraperitoneal injection of LPS in mice resulted in the upregulation of phospho-p65 compared with the controls. LFM-A13 significantly inhibited the LPS-induced phosphorylation of p65 in a dosage-independent manner. In vitro, we further used the Tec-siRNA-transfected NRK-52E cell to investigate the I*κ*B*α* phosphorylation and the degradation and phosphorylation status of p65. As shown in Figures 6(c) and 6(d), LPS enhanced the I*κ*B-*α* phosphorylation, decreased the levels of I*κ*B-*α*, and induced the phosphorylation of p65. The knockdown of Tec by si-RNA obviously abolished the phospho-p65 and I*κ*B*α* expressions in NRK-52E cells stimulated by LPS, but increased the levels of I*κ*B*α*. These data suggest that Tec kinase can be an upstream protein that leads to NF-*κ*B activation in mice after AKI.

### 3.7. TLR4 And MyD88 Are Important Upstream Proteins That Regulate the NF-*κ*B Activity

Therefore, we also examined the renal expressions of TLR4 and MyD88. As shown in Figures 6(e) and 6(f), the steady expressions of TLR4 and MyD88 in mice pretreated with LFM-A13 after injury were significantly lower than those in the AKI induced by LPS injection. Altogether, these results indicate that the inhibition of Tec kinase may suppress upstream signals and lead to the activation of NF-*κ*B after AKI.

## 4. Discussion

In the present study, LPS administration induced apparent renal injury in mice, including elevated levels of urea and Cr in plasma, an increase in plasma Cys-C, and tubular cell disruption. Serum Cys-C indicates the real-time functional state of the kidney. It has been suggested to be an endogenous marker for predicting the early and accurate diagnosis of AKI [22–24]. We observed that Cys-C was detected at high levels in LPS-exposed mice, identifying renal dysfunction in the early stages of AKI. All manifestations were significantly protected by LFM-A13 pretreatment. LFM-A13, a leflunomide metabolite analogue, has been used to inhibit Tec protein expression [15, 16]. Tec kinase has been noticed and trapped in acute inflammatory response recently. In our previous study, direct evidence that LPS stimulates an increase in the phosphorylation of Tec and total Tec protein in macrophages was obtained [16]. In this study, Tec kinase was induced in a mouse model of AKI and tubular epithelial cells exposed by LPS. In accordance with a previous study, the importance of Tec kinase as a mediator in AKI was suggested.

Tec kinase has been implicated in regulating the acute inflammatory response in several publications [25–28]. In our pervious study, high levels of Tec and phosphorylated Tec were observed in RAW263.7 macrophage exposed by LPS [16]. Gilbert has shown that Tec kinase activity was induced in human neutrophils after induction by formylmethionyl-leucyl-phenylalanine (fMLP) [29]. The present study attempted to evaluate Tec kinase in normal renal tissue and tubular cell after acute injury. Our data indicate that the activation of Tec kinase in mice after AKI is disadvantageous and causes renal damage, as tubule-specific presence of Tec protein results in renal dysfunction such as elevated serum Cr, BUN, Cys-C, and renal pathological injury after LPS administration. In AKI induced by LPS, tubular cell injury or necrosis is a major pathogenic mechanism that leads to acute renal failure [5, 30, 31]. Consistent with renal tissues, renal tubular cell, NRK-52E, exhibited Tec protein induction after LPS treatment. These results indicate that the activation of Tec kinase in renal tubules promotes the injury response of the kidneys.

LPS-induced AKI is associated with abnormal inflammatory response, including renal endothelial dysfunction and renal inflammation. Of the mechanisms, inflammation is widely accepted as an important player. Two prototypic proinflammatory TNF-*α* and IL-1*β* induced by LPS have been reported in acute inflammation, including our previous studies [32–34]. In the present study, we observed an increased TNF-*α* and IL-1*β* production and a high renal injury score. LFM-A13 exhibited an inhibitory effect on inflammatory cytokines in LPS administration. A controversy exists on the concentration of LFM-A13 for reducing cytokine production in neutrophils and macrophages [16, 29]. However, a nonlinear dosage-dependent effect of LFM-A13 was observed in this study. These findings are difficult to reconcile, and further studies are required to clarify this issue.

The present study indicates that the activation of Tec kinase may promote AKI by a multitude of mechanisms. Decreasing the Tec expression by LFM-A13 in vivo or Tec-siRNA in vitro results in the inactivation of the NF-*κ*B pathway with the evident phosphorylation of p65 and I*κ*B*α* and degradation of I*κ*B*α*. NF-*κ*B has been reported extensively as a key regulator of proinflammatory signals in various inflammatory conditions in many studies, including our previous studies [16, 35, 36]. These suggest that NF-*κ*B may have a critical role in mediating the proinflammatory effect of Tec kinase. TLR4, a member of the Toll-like receptor family of transmembrane proteins, recognizes pathogens, such as LPS, and is responsible for the inflammatory cascade in sepsis [37–39]. TLR4 can bind to its adaptor, MyD88, and participates in downstream signaling and mediates the activation of a transcriptional factor, such as NF-*κ*B, mediating the expression of proinflammatory cytokines, such as TNF-*α* and IL-1*β* [40–42]. Our previous study identified that endogenous ligands, such as LPS and high mobility group box-1 protein, can also activate the TLR4 pathway [32]. In the present study, we also demonstrated that LPS can increase the expressions of TLR4 and MyD88. To investigate whether the TLR4 and MyD88 expressions can be upregulated by Tec kinase, we pretreated mice with a Tec kinase inhibitor, LFM-A13, prior to LPS injection. The results showed that LFM-A13 can significantly inhibit the LPS-enhanced TLR4 and MyD88 expressions. The present study showed that TLR4\MyD88\NF-*κ*B is an important signaling pathway affected by Tec inhibition by LFM-A13 for attenuating LPS-induced AKI by inhibiting the inflammatory response. However, whether the other adaptor molecules or modulator participates in Tec kinase-induced transcellular signaling is unclear. The detailed mechanism for the role of Tec kinase in AKI should be clarified by further research.

## 5. Conclusions

In summary, we report herein that Tec kinase is induced in the mouse model of AKI induced by LPS. The present study evaluated the effects of LFM-A13 on LPS-induced AKI, showing the ability of LFM-A13 to attenuate the LPS-induced renal dysfunction. These findings suggest that the renal activation of Tec kinase after AKI promotes renal tubular cell injury. The protective effect of LFM-A13 or Tec-siRNA is correlated with its potential to modulate Tec kinase, downregulating the TLR4, MyD88, and NF-*κ*B pathways and decreasing the inflammatory response. Further studies are required to verify the direct molecular interaction with Tec kinase.

## Figures and Tables

**Figure 1:** LPS-induced acute kidney injury. C57BL/6 mice (male, 8–12 weeks old) were divided into 5 groups and subjected to the following treatment: (1) control (injected with saline); (2) LPS treatment for 1 h; (3) LPS treatment for 6 h; (4) LPS treatment for 24 h; (5) LPS treatment for 48 h. (a–c) Blood samples were collected for BUN, creatinine, and Cys-C measurement. (d) Representative images of HE staining of kidney tissues from control and LPS- (20 mg/kg) treated mice at 1, 6, 12, 24, and 48 h. Bar = 25 *μ*m. (e) Pathological score of representative renal tissue samples of each group. The scoring based on the area of interstitial inflammation and fibrosis, tubular atrophy, and dilation with cast formation involving percentage of the field. 0: normal; 1: <25%; 2: between 25% and 50%; 3: >50%. The score was calculated by averaging the grades assigned to all tubule fields. The data are expressed as the mean ± SEM of 5 mice in each group. ^∗^*P* < 0.05 and ^∗∗^*P* < 0.01, significant difference vs. control.

**Figure 2:** LPS-induced Tec kinase expression in kidney tissue and NRK-52E cell. (a, b) The expression of Tec kinase was detected by Western blot in LPS- (20 mg/kg) treated mice at 1, 6, 24, and 48 h. Quantitative analysis of Tec protein was determined by integral optical density (^∗∗^*P* < 0.01, ^∗^*P* < 0.05, *n* = 5). (c) Immunohistochemical analysis of Tec kinase expression in kidney tissue. Bar = 50 *μ*m. (d) The expression of Tec kinase was detected by Western blot in NRK-52E cell exposed with various concentrations of LPS (0.01, 0.1, 1, and 10 *μ*g/mL). The relative expression was quantified (^∗∗^*P* < 0.01, *n* = 5). (e) The expression of Tec kinase was detected in NRK-52E cell after 0.1 *μ*g/mL LPS stimulus at different times. The relative level of Tec kinase was quantified. 0.1 *μ*g/mL LPS increased the Tec expression in a time-dependent manner, with a peak at 60 min (^∗∗^*P* < 0.01, *n* = 5).

**Figure 3:** LFM-A13 pretreatment alleviates LPS-induced AKI. In the LPS group, mice were i.p. injected with LPS (20 mg/kg). In the LFM-A13+LPS group, mice were pretreated with LFM-A13 dose (40, 60, and 80 mg/kg) immediately after LPS injection. Blood samples and kidney tissues were collected at 24 h after LPS i.p. (a–c) Renal function including BUN, sCr, and Cys-C was measured 24 h after LPS injection. (d) Renal histopathology was evaluated 24 h after LPS injection. An obvious renal pathological damage, including tubular cell swelling, dilatation, lysis, destruction of tubular structures, and neutrophil emigration (solid arrows), was observed after LPS treatment. Bar = 50 *μ*m. (e) Pathological scores of tubular damage among different groups. All data were expressed as the means ± SEM. ^∗∗^*P* < 0.01, ^∗^*P* < 0.05.

**Figure 4:** LFM-A13 inhibited Tec protein expression in LPS-induced AKI. (a) Representative immunohistochemical staining showed renal Tec protein staining in the control, LPS group, and different concentration of LFM-A13 (40, 60, and 80 mg/kg) prior to LPS injection. Boxed areas in the cortical and medullar regions are enlarged. Arrowheads indicate renal tubules. Bar = 50 *μ*m. (b) Expression of Tec kinase in whole kidney lysates was detected by Western blot. (c) Quantitative analysis of Tec protein was determined by integral optical density (^∗∗^*P* < 0.01, *n* = 5).

**Figure 5:** The effect of LFM-A13 on TNF-*α* and IL-1*β* levels after LPS administration. Quantitation of TNF-*α* and IL-1*β* in renal tissues was measured by ELISA. All data were represented as the means ± SEM. ^∗∗^*P* < 0.01, ^∗^*P* < 0.05. *n* = 5.

**Figure 6:** Effects of LFM-A13 or Tec-siRNA on the expression of the NF-*κ*B pathway and TLR4/MyD88 in LPS-induced AKI or LPS-stimulated NRK-52E cell. Protein extracts were obtained from kidney tissues and NRK-52E cells, and protein expression level was detected by Western blot analysis. (a, b) Expressions of NF-*κ*B p65 and p-p65 in kidney tissues were analyzed by Western blot. The relative expression of p-p65 was quantified with a densitometry. LFM-A13 pretreatment inhibited the activity of NF-*κ*B p-p65. (c, d) Expressions of NF-*κ*B p65, p-p65, I*κ*B*α*, and p-I*κ*B*α* in NRK-52E cell were detected by immunoblotting. The relative levels were quantified. LPS promoted phosphorylation of NF-*κ*B p65, while Tec-siRNA protected degradation of I*κ*B*α* and inhibited phosphorylation status of p65 and I*κ*B*α*. (e, f) Expressions of TLR4 and MyD88 were detected and quantified. LFM-A13 pretreatment reduced LPS-induced TLR4/MyD88 expression. Densitometric analysis of the results expressed as arbitrary units of the mean ± SEM of each group. ^∗∗^*P* < 0.01, ^∗^*P* < 0.05. *n* = 5.

## Data Availability

All data generated or analyzed during this study are included in this published article.

## Abbreviations

AKI: Acute kidney injury
Cr: Creatinine
BUN: Blood urea nitrogen
Cys-C: Cystatin-C
LFM-A13: Leflunomide metabolite analogue
Tec: Tyrosine kinase expressed in hepatocellular carcinoma
LPS: Lipopolysaccharide
IL-1*β*: Interleukin 1*β*
TNF-*α*: Tumor necrosis factor *α*
MyD88: Myeloid differentiation factor 88
TLR4: Toll-like receptor 4
NF-*κ*B: Nuclear factor-kappa B.

## References

[1] Joannidis M., Druml W., Forni L. G. (2017). Prevention of acute kidney injury and protection of renal function in the intensive care unit: update 2017: expert opinion of the Working Group on Prevention, AKI section, European Society of Intensive Care Medicine. *Intensive Care Medicine*.

[2] Basile D. P., Bonventre J. V., Mehta R. (2016). Progression after AKI: understanding maladaptive repair processes to predict and identify therapeutic treatments. *Journal of the American Society of Nephrology*.

[3] Zarjou A., Agarwal A. (2011). Sepsis and acute kidney injury. *Journal of the American Society of Nephrology*.

[4] Ohnuma T., Uchino S. (2017). Prediction models and their external validation studies for mortality of patients with acute kidney injury: a systematic review. *PLoS One*.

[5] Zarbock A., Gomez H., Kellum J. A. (2014). Sepsis-induced acute kidney injury revisited: pathophysiology, prevention and future therapies. *Current Opinion in Critical Care*.

[6] Gomez H., Ince C., Backer D. D. (2014). A unified theory of sepsis-induced acute kidney injury. *Shock*.

[7] Ricci Z., Ronco C. (2009). Pathogenesis of acute kidney injury during sepsis. *Current Drug Targets*.

[8] Feng D., Wang Y., Liu Y. (2018). DC-SIGN reacts with TLR-4 and regulates inflammatory cytokine expression via NF-*κ*B activation in renal tubular epithelial cells during acute renal injury. *Clinical and Experimental Immunology*.

[9] Fu H., Hu Z., Di X., Zhang Q., Zhou R., Du H. (2016). Tenuigenin exhibits protective effects against LPS-induced acute kidney injury via inhibiting TLR4/NF-*κ*B signaling pathway. *European Journal of Pharmacology*.

[10] Castoldi A., Braga T. T., Correa-Costa M. (2012). TLR2, TLR4 and the MYD88 Signaling Pathway Are Crucial for Neutrophil Migration in Acute Kidney Injury Induced by Sepsis. *PLoS One*.

[11] Li F., Jiang Y., Zheng Q., Yang X., Wang S. (2011). TEC protein tyrosine kinase is involved in the Erk signaling pathway induced by HGF. *Biochemical and Biophysical Research Communications*.

[12] Cenni B., Gutmann S., Gottar-Guillier M. (2012). BMX and Its Role in Inflammation, Cardiovascular Disease, and Cancer. *International Reviews of Immunology*.

[13] Page T. H., Urbaniak A. M., Espirito Santo A. I. (2018). Bruton’s tyrosine kinase regulates TLR7/8-induced TNF transcription via nuclear factor-*κ*B recruitment. *Biochemical and Biophysical Research Communications*.

[14] Tampella G., Kerns H. M., Niu D. (2015). The Tec kinase-regulated phosphoproteome reveals a mechanism for the regulation of inhibitory signals in murine macrophages. *The Journal of Immunology*.

[15] Zemans R. L., Arndt P. G. (2009). Tec kinases regulate actin assembly and cytokine expression in LPS-stimulated human neutrophils via JNK activation. *Cellular Immunology*.

[16] Wang F., Zhang W., Wang C. (2017). Inhibitor of Tec kinase, LFM-A13, decreases pro-inflammatory mediators production in LPS-stimulated RAW264.7 macrophages via NF-*κ*B pathway. *Oncotarget*.

[17] Schwalm S., Beyer S., Frey H. (2017). Sphingosine kinase-2 deficiency ameliorates kidney fibrosis by up-regulating Smad 7 in a mouse model of unilateral ureteral obstruction. *The American Journal of Pathology*.

[18] Tavares M. B., Almeida M. d. C. C. d., Martins R. T. C., de Sousa A. C. G. P., Martinelli R., dos-Santos W. L. C. (2012). Acute Tubular Necrosis and Renal Failure in Patients with Glomerular Disease. *Renal Failure*.

[19] Dai X., Zeng Z., Fu C., Zhang S.’a., Cai Y., Chen Z. (2015). Diagnostic value of neutrophil gelatinase-associated lipocalin, cystatin C, and soluble triggering receptor expressed on myeloid cells-1 in critically ill patients with sepsis-associated acute kidney injury. *Critical Care*.

[20] Shi M., Zeng X., Guo F. (2017). Anti-inflammatory pyranochalcone derivative attenuates LPS-induced acute kidney injury via inhibiting TLR4/NF-*κ*B pathway. *Molecules*.

[21] Tarantino N., Tinevez J. Y., Crowell E. F. (2014). TNF and IL-1 exhibit distinct ubiquitin requirements for inducing NEMO-IKK supramolecular structures. *The Journal of Cell Biology*.

[22] Kar S., Paglialunga S., Islam R. (2018). Cystatin C is a more reliable biomarker for determining eGFR to support drug development studies. *The Journal of Clinical Pharmacology*.

[23] Teo S. H., Endre Z. H. (2017). Biomarkers in acute kidney injury (AKI). *Best Practice & Research. Clinical Anaesthesiology*.

[24] Bagshaw S. M., Bellomo R. (2010). Cystatin C in acute kidney injury. *Current Opinion in Critical Care*.

[25] Broides A., Hadad N., Levy J., Levy R. (2014). The Effects of Bruton Tyrosine Kinase Inhibition on Chemotaxis and Superoxide Generation in Human Neutrophils. *Journal of Clinical Immunology*.

[26] Liu C. C., Lai C. Y., Yen W. F. (2015). Reciprocal Regulation of C-Maf Tyrosine Phosphorylation by Tec and Ptpn22. *PLoS One*.

[27] Zwolanek F., Riedelberger M., Stolz V. (2014). The Non-receptor Tyrosine Kinase Tec Controls Assembly and Activity of the Noncanonical Caspase-8 Inflammasome. *PLoS Pathogens*.

[28] Koprulu A. D., Ellmeier W. (2009). The role of Tec family kinases in mononuclear phagocytes. *Critical Reviews™ in Immunology*.

[29] Gilbert C., Levasseur S., Desaulniers P. (2003). Chemotactic Factor-Induced Recruitment and Activation of Tec Family Kinases in Human Neutrophils. II. Effects of LFM-A13, a Specific Btk Inhibitor. *The Journal of Immunology*.

[30] Kosaka J., Lankadeva Y. R., May C. N., Bellomo R. (2016). Histopathology of septic acute kidney injury: a systematic review of experimental data. *Critical Care Medicine*.

[31] Moeckel G. W. (2018). Pathologic perspectives on acute tubular injury assessment in the kidney biopsy. *Seminars in Nephrology*.

[32] Chen X. L., Sun L., Guo F. (2012). High-Mobility Group Box-1 Induces Proinflammatory Cytokines Production of Kupffer Cells through TLRs-Dependent Signaling Pathway after Burn Injury. *PLoS One*.

[33] Guo F., Chen X. L., Wang F., Liang X., Sun Y. X., Wang Y. J. (2011). Role of Angiotensin II Type 1 Receptor in Angiotensin II-Induced Cytokine Production in Macrophages. *Journal of Interferon & Cytokine Research*.

[34] Wang F., Xia Z. F., Chen X. L., Jia Y. T., Wang Y. J., Ma B. (2009). Angiotensin II type-1 receptor antagonist attenuates LPS-induced acute lung injury. *Cytokine*.

[35] Fang H., Jiang W., Cheng J. (2015). Balancing innate immunity and inflammatory state via modulation of neutrophil function: a novel strategy to fight sepsis. *Journal of Immunology Research*.

[36] Tongaonkar P., Trinh K. K., Schaal J. B. (2015). Rhesus macaque *θ*-defensin RTD-1 inhibits proinflammatory cytokine secretion and gene expression by inhibiting the activation of NF-*κ*B and MAPK pathways. *Journal of Leukocyte Biology*.

[37] Schappe M. S., Szteyn K., Stremska M. E. (2018). Chanzyme TRPM7 mediates the Ca^2+^ influx essential for lipopolysaccharide-induced Toll-like receptor 4 endocytosis and macrophage activation. *Immunity*.

[38] Plociennikowska A., Hromada-Judycka A., Borzecka K., Kwiatkowska K. (2015). Co-operation of TLR_4_ and raft proteins in LPS-induced pro-inflammatory signaling. *Cellular and Molecular Life Sciences*.

[39] Ryu J. K., Kim S. J., Rah S. H. (2017). Reconstruction of LPS transfer cascade reveals structural determinants within LBP, CD14, and TLR4-MD2 for efficient LPS recognition and transfer. *Immunity*.

[40] Xu M. X., Wang M., Yang W. W. (2017). Gold-quercetin nanoparticles prevent metabolic endotoxemia-induced kidney injury by regulating TLR4/NF-*κ*B signaling and Nrf2 pathway in high fat diet fed mice. *International Journal of Nanomedicine*.

[41] Pan Q., Zhang Q., Chu J. (2017). *Chlamydia abortus* Pmp18.1 induces IL-1*β* secretion by TLR4 activation through the MyD88, NF-*κ*B, and caspase-1 signaling pathways. *Frontiers in Cellular and Infection Microbiology*.

[42] Cong L., Yang S., Zhang Y., Cao J., Fu X. (2018). DFMG attenuates the activation of macrophages induced by co‑culture with LPC‑injured HUVE‑12 cells via the TLR4/MyD88/NF‑*κ*B signaling pathway. *International Journal of Molecular Medicine*.

